The article "Improvements of Physical Activity Performance and Motivation in Adult Men through Augmented Reality Approach: A Randomized Controlled Trial" was published in 2022. Journal: J Environ Public Health.

# Improvements of Physical Activity Performance and Motivation in Adult Men through Augmented Reality Approach: A Randomized Controlled Trial

**DOI:** 10.1155/2022/3050424

**Published:** 2022-07-09

**Authors:** Daekook M. Nekar, Hye Yun Kang, Jae Ho Yu

**Affiliations:** Department of Physical Therapy, Sunmoon University, Asan-si, Republic of Korea

## Abstract

The COVID-19 pandemic had a global impact, increasing the prevalence of physical inactivity, which is mostly due to the lockdown and social distancing measures adopted during the pandemic. Hence, this study aimed to compare the efficacy of augmented reality-based training on physical activity performance and motivation in healthy adults to mirror visual feedback training and conventional physical therapy. This study used the randomized control trial pretest-posttest research design. Forty-eight healthy men aged 18–35 years who were engaged in recreational physical activities were enrolled and randomly divided into four groups: augmented reality-based training reality (ART), mirror visual feedback training (MVFT), therapist-based training (TBT), and control group. The total training program was held for four weeks. The isokinetic dynamometer, sit-and-reach test, Y balance test, and the intrinsic motivation inventory-22 were used to measure the outcomes before and after the intervention. Paired sample *t*-test was used to compare the changes before and after the intervention within groups, while the one-way ANOVA was used for the comparison between the groups. Results of the study showed that, after four weeks of intervention, balance, muscle strength, and muscle endurance in all groups significantly improved except for the control group. The ART group showed the highest increase in muscle strength, muscle endurance, and balance compared to the other groups. The motivation level increased in all three feedback groups and was observed in the following order: ART group > MVFT group > TBT group > control group. This study highlighted the most effective method that may be applied for home training during and after this period of the pandemic. The findings revealed that training while receiving real-time feedback via AR devices improves both physical performance and motivation. Augmented reality-based training can be used as an effective training option for improving physical activity and motivation and can be suggested for home training programs.

## 1. Introduction

The novel coronavirus outbreak, otherwise known as COVID-19, was firstly identified in Wuhan, China, then rapidly spread worldwide, and has been declared in March 2020 by the World Health Organization as a pandemic [1]. The COVID-19 pandemic has severely affected the economy, social interactions, and daily activities of people around the world. Furthermore, the lockdown and social distancing measures used in many countries to prevent the spread of the virus caused anxiety and stress and negatively influenced population's daily routines, behavior, and physical activity [2]. Compared to the prepandemic situation, most outdoor facilities such as fitness centers become empty or closed because people avoid public/enclosed spaces. During this period of the pandemic, maintaining a strong immune system is crucial to improve the ability to fight against the virus infection and limit the severity of the symptoms in case of infection [3].

The article "Improvements of Physical Activity Performance and Motivation in Adult Men through Augmented Reality Approach: A Randomized Controlled Trial" was published in 2022. Journal: J Environ Public Health.

Physical activity is widely known for its benefits on health, and numerous studies support this fact. Consistent physical activity is a key factor in reducing the risk of numberless persistent diseases associated with the risk of death [4, 5]. According to previous studies, physical exercise operates as a regulator that significantly strengths the immune system and promotes a better quality of life [6, 7]. Moreover, a recent study revealed that physical activity is fundamental in lowering the risk of severe COVID-19 infection in persons who are infected [8]. However, despite all the positive impacts of physical activity, the number of insufficiently active people remains significant, and sedentary life (lack of physical activity) is one of the serious health issues of the twenty-first century [4, 9]. The World Health Organization reported since 2016 that 23% of men and 32% of women did not complete the recommendations for physical activity and around 81% of adolescents were not sufficiently active [10]. According to the report of the Ministry of Culture, Sport and Tourism of Korea, the Korean population's lifestyle has suddenly changed since the beginning of the pandemic, and particularly, the level of physical activity has reduced from 66.6% in 2019 to 60.1% in 2020 and may continue to decrease [11]. Due to the restricted outdoor mobility and accessibility of sports facilities, home training can be considered as a potential adequate alternative solution to help people maintain normal fitness levels/physical activity and reduce psychosocial and all related health issues.

However, a continuous and adequate stimulation maintaining the level of interest in the activity is primordial to enhance physical activity participation and expect beneficial results. Many types of feedback such as therapist-based feedback, mirror visual feedback, and innovative technologies using augmented reality (AR) or virtual reality-based training are being used in the rehabilitation and sports field to improve performance [12–14]. Several studies have reported the effectiveness of therapist-based feedback in improving physical activity, while also maintaining motivation and self-confidence in junior athletes [14, 15]. This method is the standard and most used feedback method during physical training in healthcare facilities and sports clubs.

The article "Improvements of Physical Activity Performance and Motivation in Adult Men through Augmented Reality Approach: A Randomized Controlled Trial" was published in 2022. Journal: J Environ Public Health.

Mirror visual feedback training (MVFT) is another form of feedback that is a well-known method used for hand and upper extremity rehabilitation in hemiplegic patients. Previous studies have reported its benefits on hand function, motor performance, and balance ability in patients with stroke and for postural control in healthy individuals [16–18]. Generally, in fitness clubs or sports centers (e.g., dancing centers), exercises are performed in front of mirrors. Receiving visual and proprioceptive feedback through the body mirroring effect may be beneficial as a means of facilitating activity performance and stimulating motivation. However, no study has evaluated the potential effect of mirror visual feedback on healthy people specially to facilitate motivation and improve physical activity performance such as balance, flexibility, strength, and endurance.

Modern devices using virtual reality and augmented reality (AR) technology have been developed, and the market is increasing. Devices using this modern technology have been reported effective to increase academic motivation and physical activity participation [19, 20]. Training using AR which provides real-time feedback increases self-motivation and encouragement of patients with cerebral vascular diseases [19]. Khan et al. [20] showed that the application of AR improved the motivation of learning and academic achievement of students. Recently, AR can be easily accessed through divers' innovative methods such as mobile phones, wearable devices, and computers [21]. According to the existing evidence, physical activity and motivation can be improved through AR devices. This method of training can be used by individuals for home training without the supervision of a health professional and can be easily applied in this period of pandemic during which outdoor mobility is limited. However, no prior research assessed the efficacy of AR-based training on motivation and physical performance for a home training physical activity program in healthy people. Moreover, no previous study has compared the effectiveness of the different training feedback (therapist-based training, mirror visual feedback training, and AR-based training) on muscle strength, muscle endurance, balance, flexibility, and motivation. Thus, it remains unclear whether the AR-based training is more effective than the therapist-based feedback and mirror visual feedback for improving physical activity performance and motivation of healthy people during self-training or home training.

The article "Improvements of Physical Activity Performance and Motivation in Adult Men through Augmented Reality Approach: A Randomized Controlled Trial" was published in 2022. Journal: J Environ Public Health.

Therefore, the goal of this research was to compare the effectiveness of augmented reality-based training on physical activity performance (muscle strength, endurance, balance, and flexibility) and motivation in healthy recreational adults to mirror visual feedback training, conventional physical therapy, and a control group. This study tends to highlight whether using AR devices that provide real-time audiovisual feedback is more effective than feedback provided by a therapist or mirror visual feedback. The findings of this study would provide evidence on the effective method that can be used to improve physical activity performance and motivation during and after the COVID-19 pandemic.

This study hypothesizes that AR-based training will improve all the target outcomes while being superior to or comparable to therapist-based training. Second, while mirror visual feedback training would enhance all the outcomes, it would be comparable to or inferior to therapist-based training and AR-based training. The present study aimed to compare the effectiveness of augmented reality-based training on physical activity performance (muscle strength, endurance, balance, and flexibility) and motivation in healthy recreational adults to mirror visual feedback training, conventional physical therapy, and a control group.

## 2. Theoretical and Conceptual Framework

### 2.1. Physical Activity Performance

Physical activity performance can be defined as the ability to execute physical activities (e. g., leisure activities, transportation, and activities of daily living) [22]. Several factors such as strong muscle strength and muscle endurance, stable balance ability, and good flexibility contribute to improving physical activity performance.

- Muscle strength: the amount of force a muscle can produce with a single maximal effort
- Muscle endurance: the ability to produce and sustain muscle force over a certain period
- Balance: the ability to maintain the line of gravity within the base of support
- Flexibility: the ability of muscles and joints to move through an unrestricted, pain-free range of motion

Greater muscle strength is identified as the factor that enhances mechanical power and reduces the risk of injury during the performance of physical activity [23]. Higher muscle endurance increases the ability to resist against muscle fatigue and allows the performance of the physical activity for a long period [24]. Flexibility and balance reduce the risk of muscle spasms and injury and increase physical activity performance [24]. Interestingly, Kartal [25] reported a relationship between flexibility and balance with optimum flexibility leading to a higher balance ability. The author also mentioned a positive relationship between muscle strength and balance with greater muscle strength and higher balance ability [25]. Various exercise methods are used according to the specific field of training to increase muscle strength, muscle endurance, flexibility, and balance ability.

The article "Improvements of Physical Activity Performance and Motivation in Adult Men through Augmented Reality Approach: A Randomized Controlled Trial" was published in 2022. Journal: J Environ Public Health.

### 2.2. Feedback and Motivation

Performance of exercise during training sessions requires sufficient motivation. Motivation is an individual's inner will to reach a particular goal and can be considered the key factor of training since it allows individuals to exercise more than their usual capacity [26]. Feedback is an essential element that is being used for increasing motivation. It can be provided through visual observation or verbal instruction. There are several theories on which feedback may have different effects on motivation according to how it is provided and how the individual understands the feedback signal. There is a theory that visual observation combined with verbal instruction had a better outcome compared to single feedback on the performance of physical activities [27]. However, another theory suggested single feedback using visual observation had more benefits than verbal instruction [28]. More interestingly, the type of visual observation may lead to a desperate effect on motivation. There is a theory that observing a demonstration made by a professional had more positive effects on motivation compared to a demonstration made by a peer or self-observation [29]. In the present study, we used the above three theories in the intervention method with feedback provided by an AR device, a therapist, and a mirror.

### 2.3. Types of Feedback Approaches

#### 2.3.1. Augmented Reality-Based Training

AR-based training refers to the application of interactive digital elements via various platforms such as Wii and Xbox. The AR exercise program provides instructions on the ongoing movement and can track the user's movement and adjust or repeat the movements. The AR-based training provides feedback in the form of visual observation with a demonstration of the exercise by an expert model. Additionally, it provides verbal cues which correspond to the verbal instruction feedback theory. Moreover, the AR-based training corresponds also to the combined visual and verbal feedback approach. This method of training has been used for different purposes including physical activity, psychology, and physical performance training in both healthy individuals and patients [30]. Research revealed the effectiveness of the above AR concepts of feedback training. For time being, it seems ideal to integrate the AR with a simple exercise and compare it to a combined visual and verbal feedback without an expert demonstration (therapist-based training) and to single visual feedback with self-observation (mirror visual feedback).

The article "Improvements of Physical Activity Performance and Motivation in Adult Men through Augmented Reality Approach: A Randomized Controlled Trial" was published in 2022. Journal: J Environ Public Health.

#### 2.3.2. Therapist-Based Training

Therapist-based training (TBT) is the basic method of patient and therapist training session in which the therapist supervises and coaches the ongoing training, gives instructions to correctly perform the movements, and improves the skills of the task. This method of providing feedback corresponds to a combined visual and verbal feedback approach mentioned above. Previous research revealed that continuous therapist feedback is effective in improving the physical condition of patients and reduces the intervention period. For example, Knittle et al. [31] reported increases in physical activity performance time after the therapist-based intervention to improve physical activity among patients with rheumatoid arthritis. Equivalent results were found by O'Halloran et al. [32] who examined the effects of therapist-based training on patients with hip fractures. Additionally, recent studies affirmed that verbal and nonverbal coaching/feedback plays a significant role in improving the self-determination and motivation of healthy athletes [33, 34].

#### 2.3.3. Mirror Visual Feedback Training

Mirror visual feedback training (MVFT) was applied firstly as a psychophysiological therapy in 1995 for amputated patients and uses the mirror-reflected image to train a specific part of the body [35]. It has also been used for patients with brain disorders (e. g., stroke and cerebral palsy) [12]. Nowadays, it is a favorable approach used to improve the physical performance of patients and healthy individuals. Previous studies used different types of exercises such as hand rotation and finger combined movement in healthy individuals and reported better physical performance after MVFT [36, 37].

## 3. Methods

### 3.1. Research Design

This study was a randomized control trial pretest-posttest design conducted on healthy adult males at Sunmoon University. The study respondents were randomly allocated to four different groups and participated in an intervention program of four weeks with outcome measurements conducted before and after the intervention. The study procedure was conformed to the Declaration of Helsinki, approved by the Institutional Review Board of Sunmoon University (SM-202104-029–2), and was registered at the Clinical Research Information Service-Korea (CRIS: KCT0006907). Before being involved in the experimental procedure, all the respondents were entirely instructed about the goal of the study and provided written consent for participation. All the research procedure was conducted in the research laboratory of the Department of Physical Therapy, Sunmoon University, by trained physical therapists.

The article "Improvements of Physical Activity Performance and Motivation in Adult Men through Augmented Reality Approach: A Randomized Controlled Trial" was published in 2022. Journal: J Environ Public Health.

### 3.2. Sample Size Calculation

For the current study, the sample size calculation was done using the computer software G∗power version 3.1.9.7 (Heinrich Heine, University, Düsseldorf, Germany). We considered an effect size of 0.25 with an alpha level (type I error) of 0.05, four groups, and five measurements. Based on these values, a sample size of 48 respondents was needed to achieve 95% of the power. Knowing that 48 respondents were the required sample size for this study, we used a mixed controlled quota and voluntary response sampling method. The use of the mentioned two methods of sampling was to recruit volunteer respondents who were eligible to participate in this study to represent our targeted population according to the inclusion criteria predefined.

### 3.3. Respondents of the Study

Respondents of the study were forty-eight men aged between 18 and 35 years old engaged in recreational physical activities. Individuals with no physical disease, no mental depression or related mental diseases, and no social problems were defined as healthy. A brief interview was conducted during the recruitment process to assess the eligibility of the respondents. Respondents who engaged in moderate-intensity aerobic physical activity at a minimum of 100 minutes per week or muscle-strengthening exercise at least once a week were included. However, those who had undergone treatment or surgery on the ankle, knee, or hip joint in the previous six months, those who have inflammation or degenerative joint disease, and those with mental illness and social problems were excluded from this study.

### 3.4. Randomization

Respondents were assigned randomly to one of the four groups: (1) group A (training with mirror visual feedback, *n* = 12); (2) group B (training while receiving verbal feedback from a physical therapist, *n* = 12); (3) group C (training and receiving feedback via an augmented reality device, *n* = 12); (4) group D (control group *n* = 12). The allocation was conducted by an independent investigator who generated 48 cards with four different colors (blue for group A, green for group B, black for group C, and yellow for control group D). The cards were put into sealed envelopes, and respondents were instructed to pick one of the 48 cards and give it to the investigator who classified each participant according to their allocated group. Respondents were blinded about the type of exercise feedback and trained in separate group training sessions.  Figure 1 presents the study's procedure flow diagram.

The article "Improvements of Physical Activity Performance and Motivation in Adult Men through Augmented Reality Approach: A Randomized Controlled Trial" was published in 2022. Journal: J Environ Public Health.

### 3.5. Outcome Measures

After allocation to respective groups, respondents' height and weight data were collected using the body part analyzers InBody 570 (Biospace, Korea) which is based on bioelectric impedance measurement (BIA). The demographic information of the respondents is presented in Table 1.

#### 3.5.1. Muscle Endurance

The knee flexion and extension muscle endurance were measured by the isokinetic dynamometer (Humac Norm Testing, CSMi, Stoughton, MA). Before the beginning of the test, respondents completed a 5-minute warm-up on a cycle ergometer with a cadence of 70–80 revolutions per minute followed by stretching to avoid injury. The manufacturer's specification was used as a reference for the calibration [38]. Respondents' upper limbs were stably strapped to the backrest of the chair to minimize compensatory movements. To familiarize themselves with the equipment and the test procedure, respondents were instructed to perform three submaximal trial repetitions before the test. The concentric endurance test included 15 maximal isokinetic knee flexion and extension of the dominant leg with knee range of motion set from 0° to 95°. Respondents were instructed to contract for 3 seconds, with a 5-second rest period between each repetition, and the investigator provided verbal encouragement to ensure respondents were contracting with the maximal force and the appropriate time. We used the fatigue index (1st peak torque (PT) minus the last (15th) PT, divided by the 1st PT multiplied by 100] to determine the muscle endurance.

#### 3.5.2. Muscle Strength

The muscle strength was assessed by the isokinetic dynamometer (Humac Norm Testing, CSMi, Stoughton, MA), which has a good and reliable tool, with ICC between 0.74 and 0.89 for knee tests [39]. The axis was aligned according to the knee joint axis. The same disposal taken for the muscle endurance test was applied to reduce compensatory irrelevant movements of the body at the moment of the test. The resistance was applied at the 1/3 distal part 2 cm above the lateral malleolus. Respondents were engaged in three submaximal isokinetic contractions at the speed of 60°/s between the range 0° to 95° with the highest peak torque (Nm) used as the maximal isokinetic strength.

#### 3.5.3. Flexibility

The sit-and-reach test was used to measure the hamstring muscle flexibility. After a proper warm-up, respondents were told to sit down with both legs straightened without shoes and with their feet against the measuring box. They were asked to put their hand together (one above another), extend their arm on the measuring box, and reach forward as far as possible with their knees extended. The measurement was performed twice with a one-minute recovery time, and the higher score was chosen.

The article "Improvements of Physical Activity Performance and Motivation in Adult Men through Augmented Reality Approach: A Randomized Controlled Trial" was published in 2022. Journal: J Environ Public Health.

#### 3.5.4. Balance

The balance was assessed through the Y balance test which is a measurement tool used to measure dynamic balance with three components (anterior, posteromedial, and posterolateral direction). It has an intrarater reliability with ICC = 0.85–0.91 and interrater reliability with ICC = 0.99–1.00 [40]. The test was conducted barefoot with the preferred leg as the stance leg. Before testing, respondents' leg length was measured, and they were asked to perform two trial tests in each direction to be familiar with the testing procedure. They were instructed to stand on the midpoint of the plate with the dominant leg and to push the yardstick far away as possible with the opposite leg. The test was conducted in the following order: anterior, posteromedial, and posterolateral, with two trials in each direction and ten seconds of rest between trials. The test was dropped out and retaken if the participant (i) could not keep the supporting foot to the center plate or touch the floor with the reaching foot or could not maintain the start and return position for one second. The best score in each direction was recorded, and the composite score, which is the addition of the three reach distances divided by three times limb length and multiplied by 100, was used for the analysis.

#### 3.5.5. Motivation

In the present study, we used the 22-item Intrinsic Motivation Inventory (IMI-22) to assess motivation in physical activity performance. The IMI-22 is the condensed version of the original 45-item scale, which was used to assess respondents' subjective experience with a specified activity. It consists of four subscales: interest/enjoyment, perceived choice, perceived competence, and pressure/tension [41]. It is evaluated on a 7-point scale with a high score designing a high level of motivation. In this study, the data were analyzed using the sum of the 22-item scores.

### 3.6. Intervention Procedure

The training program in this study consisted of four sets of squats with 30 repetitions per set and two minutes of rest between each set. The program was held three times a week for four weeks, for 12 sessions.

#### 3.6.1. Augmented Reality-Based Training Group

In this study, the mobile AR device (UINCARE-82) manufactured by UINCARE (Korea) was used for the AR-based training group. The program runs on windows and is connected to a Kinect camera v2. The exercise protocol (number of sets and repetitions) was directly programmed into the device, and respondents followed the cadence of accompanying by audio and visual correctional feedback provided after each repetition to guide movements as they exercised.

The article "Improvements of Physical Activity Performance and Motivation in Adult Men through Augmented Reality Approach: A Randomized Controlled Trial" was published in 2022. Journal: J Environ Public Health.

#### 3.6.2. Mirror Visual Feedback Group

Before beginning the program, respondents were given verbal instructions on how to perform the squat properly. The instruction was as follows: keep your feet in the middle of the hip and shoulder range, along with toes moderately rotated out (5 ∼ 15°); maintain your back in a neutral position; shoulders, back, and chest open with heels touching the floor and positioned in the direction of the move; and hands crossed in front of the chest to maintain the balance. Begin the task by sending your hip back as you are sitting back on a chair, then bend your knees downward with your chest lifted in a controlled movement. The exercises were performed in front of a whole-body mirror, with respondents adjusting their movements based on the reflected image on the mirror. The instructors did not provide them with any additional feedback.

#### 3.6.3. Therapist-Based Feedback Group

Respondents allocated to the therapist-based training group received the same instruction given to those in the MVFT group while receiving real-time correctional verbal feedback on the ongoing exercise and encouragement from the instructor.

#### 3.6.4. Control Group

Respondents in the control group received the same instruction on squat performance provided to the other groups. However, the exercise was performed in a nonmirrored experiment room, in front of a blank wall, and without any feedback provided.

### 3.7. Data Analysis

For the statistical analysis, the IBM SPSS software version 25.0 for windows (SPSS Inc, Chicago, IL, USA) was used, and the data are presented as mean ± standard deviation. A descriptive statistic was used to analyze the general characteristic of participants. The Shapiro–Wilk test was used to analyze the normality of demographic data and the outcome variables. The normality test was conducted by ordering and standardizing the sample with a 95% degree of confidence. The paired sample *t*-test was conducted to compare the within-group difference by disposing the mean variables of the pretest and posttest and analyzing the difference between the paired mean variables. The one-way ANOVA was used to analyze the difference between the groups by comparing the mean variables of the four groups. Moreover, to find out exactly which groups are different from each other, we conducted the post hoc test using the Tukey HSD test by comparing all possible pairs of means. Additionally, to quantitatively measure the magnitude of intervention methods, the effect size was calculated with the mean score difference divided by the baseline standard deviation as performed in previous studies. The effect size interpretation was small if *d* = 0.2, medium if *d* = 0.5, and large if *d* = 0.8. The significance level was set at *P* < 0.05.

The article "Improvements of Physical Activity Performance and Motivation in Adult Men through Augmented Reality Approach: A Randomized Controlled Trial" was published in 2022. Journal: J Environ Public Health.

## 4. Results and Discussion

Data were collected at the baseline before the training and at the end of the four weeks, and all respondents shared similar demographic characteristics (Table 1). Forty-eight respondents were divided equally 12 each into the four groups (ART group, MVFT group, TBT group, and control group). There was no drop-out during the entire process, and data of all respondents were analyzed and reported in the results.

Regarding the physical activity performance, there were various changes before and after the intervention. First, the knee extension and flexion strength, along with muscle endurance showed a significant increase during the pretest-posttest comparison in all the three feedback training groups (MVFT group, TBT group, and ART group) with *P* < 0.05. No improvement was observed in the control group between the pretest-post comparison (*P* > 0.05).

Second, the between-group comparison of knee extension muscle, strength, and endurance showed a significant difference between the ART group and MVFT group, between the ART group and control group, and between the TBT group and control group (*P* < 0.05) with small to very large effect size. However, no significant difference was observed between the MVFT group and the TBT group and between the MVFT group and the control group (*P* < 0.05). The comparison between groups of knee flexion muscle strength and endurance showed that the ART group and TBT group were significantly different from the control group (*P* < 0.05). However, no significant difference was observed between the three feedback training groups and between the MVFT group and the control group (*P* > 0.05). The effect size ranged from small to very small size (Table 2) (Figure 2). The result reveals a superior effect of ART followed, respectively, by the TBT and MVFT for improving muscle strength and endurance.

Third, during the comparison of balance ability between pre- and posttest, significant improvement was observed in all groups (*P* < 0.05) except the control group which did not show a statistical difference between before and after the training (*P* > 0.05) (Table 3) (Figure 3).

The between-group comparison showed that the ART group and TBT group were both significantly different compared to the control group (*P* < 0.05). There were significant differences between the TBT group and MVFT group (*P* < 0.05) and between the ART group and MVFT group (*P* < 0.05). However, no significant difference was observed between the ART group and TBT group and between the MVT group and control group (*P* > 0.05). The result revealed that training with feedback provided by a therapist and through an AR device has a similar efficacy which is superior to the MVFT.

The article "Improvements of Physical Activity Performance and Motivation in Adult Men through Augmented Reality Approach: A Randomized Controlled Trial" was published in 2022. Journal: J Environ Public Health.

Regarding flexibility, there was no statistically significant difference in the sit and reach test during the pretest-posttest in all four groups (*P* > 0.05). Moreover, the between-group comparison did not show any difference between all the groups (*P* > 0.05), and the effect size was very small for all the different training feedbacks.

After completing the feedback training program, the intrinsic motivation significantly increased from preintervention to postintervention for the ART group, TBT group, and MVFT group with *P* < 0.05 and medium to large effect size. However, the control group did not show significant improvement from pretest to posttest with *P* > 0.05. There was no significant difference between all the groups, but the effect size of each training feedback showed the improvement of motivation in the following order ART group > MVFT group > TBT group > control group (Table 3) (Figure 3). This result reveals that using AR for training provides adequate feedback to effectively improve motivation compared to the mirror visual feedback and the feedback provided by a therapist.

The current study compared the effects of three different training approaches on intrinsic motivation, muscle strength, endurance, balance, and flexibility in healthy adult males: augmented reality-based training, training supervised directly by a therapist, and mirror visual feedback training. The optimal outcome of this experiment would be that providing adequate feedback may improve motivation for sports participation, thus improving physical performance. The findings partially supported our hypotheses with an improvement in balance ability, muscle endurance, muscle strength, and motivation to participate in sports activity after training with all three feedback methods. However, the flexibility did not show significant changes regardless of the feedback method.

Repetition of limb movement over time with a sufficient load is a crucial factor in improving muscle strength and endurance. However, improvement of flexibility requires holding the technique for at least 10 seconds. In this study, hamstring flexibility did not show any significant improvement in any of the groups, regardless of the type of the provided feedback. This result may be explained by the fact that respondents performed only one exercise type which was the squat exercise. The squat is a common and popular exercise performed by a wide range of populations. It has been reported to be an effective exercise that increases muscular strength of the lower extremity and reduces possible joint injury or strain [42]. The hamstring muscles which are involved during the squat exercise play the role of knee flexor and cocontraction with the quadriceps muscles during knee extension. Therefore, we can assume that, as a muscle-strengthening exercise, squatting may reduce the range of motion and limit the flexibility of the hamstring muscles. A similar result was found in a previous study showing reduced flexibility of hamstring muscle during a heavy back squat (90–95% of 1RM) and no effect during moderate intensity (60–65% of 1RM) [43].

The article "Improvements of Physical Activity Performance and Motivation in Adult Men through Augmented Reality Approach: A Randomized Controlled Trial" was published in 2022. Journal: J Environ Public Health.

During home training or center self-training, encouragement and motivation are primordial elements for maintaining constant interest for a long time and continuous training program. Training in front of a mirror is a common method used for patients with brain injuries such as stroke patients. The findings showed that performing physical exercise while receiving direct visual feedback through a mirror improved balance, knee flexion, and extension of isokinetic muscle strength and endurance in healthy adults after four weeks. However, the obtained result was inferior compared to the auditory feedback provided by the therapist and the mixed auditory-visual feedback provided through the AR device. This result is similar to a previous study conducted by Yang et al. [44] on patients with Pusher syndrome. They affirmed improvement of balance and lower extremity control through mirror visual feedback but inferior to computer interactive feedback. Authors explained this difference by the fact that mirror visual feedback is unable to provide quantified data which may enhance encouragement and motivation. The common feedback receptors during the motor learning process are the eyes, ears, and skin. Visual feedback has been reported to provide messages regarding the body/object locations in space and is effective for movement correction [45]. However, with the mirror visual feedback, respondents receive limited information (only visual cues), and they report feeling no enjoyment during the sessions.

In the present study, the auditory feedback provided by the therapist was effective to improve motivation and physical performance. Respondents' personalities and therapist characteristics are part of the factors influencing self-motivation [46]. Thus, we assume that the presence of the therapist can allow psychological self-confidence and encouragement as a placebo effect. Auditory feedback provided is considered a useful source of additional information when the visual system is overloaded [47]. Additionally, providing information, having a good rapport, and chatting with patients can stimulate motivation [48]. In this study, the therapist did not only provide correctional feedback but additionally provided encouragement and count the number of the squat exercise on a rhythmic sequence allowing respondents to maintain a constant rhythm and self-determination.

The article "Improvements of Physical Activity Performance and Motivation in Adult Men through Augmented Reality Approach: A Randomized Controlled Trial" was published in 2022. Journal: J Environ Public Health.

Feedback provided by the augmented reality device presented better improvement in balance, muscle strength, muscle endurance, and motivation after the 4 weeks of the training program in the present study. This result is consistent with a previous study with computer-generated interactive visual feedback [44]. The interactive visual feedback provided more information such as quantified data which is not possible with the other feedback methods. The augmented reality device used in the present study can not only provide visual information to correct position during the exercise but also special effects after each repetition of the exercise helping to enhance the interest in the ongoing task. Despite the visual feedback, augmented reality provides real-time auditory feedback keeping the respondents concentrate and determine to pursue the next repetition. Additionally, the training via the augmented reality device provides a score on the accuracy of the task and time of the performance which respondents tried to maintain the highest score. Zhu et al. [47] affirmed that knowing the result leads to a self-determination to do better than the last score which stimulates motivation. Thus, self-determination may be the main reason for the superiority of augmented reality feedback. This explanation is supported by a previous study affirming that goal-oriented tasks and knowledge of the performance are fundamental factors for increasing interest and motivation for the ongoing task [49–52]. Moreover, respondents in the present study reported that the combination of the real world along with virtual objects, providing a joined real and the virtual environment kept them attracted to the exercise content. With the development of technology, augmented reality/virtual reality can be easily accessed through smartphones or tablets using android at a low price. Training while receiving feedback from an augmented reality device or mobile phone-based augmented reality can be suggested for continuous self-training/home training.

## 5. Conclusion

The present study aimed to compare the efficacy of augmented reality-based training on physical activity performance and motivation in healthy adults to mirror visual feedback training and conventional physical therapy. The augmented reality-based training has more efficacy in improving balance, muscle strength, muscle endurance, and motivational level compared to the mirror visual feedback training and therapist-based training. However, the present study has some limitations that need to be acknowledged. First, the study focused only on the type of different feedback with only one exercise targeting the lower extremity. Secondly, the intervention was conducted for 4 weeks without a follow-up on respondents to monitor and assess the long-term effect on the motivation outcome. Moreover, the result cannot be generalized since all respondents included in the experiment were only adult males. Further study is needed to evaluate the effects of diverse types of exercises in the long term and provide more evidence on the topic. Despite the above limitations, the present study provides insights to effectively increase and maintain normal physical activity and motivation in this time of COVID-19 during which people present limited mobility and decreased physical activity. With the findings of this study, we can suggest the use of augmented reality-based training for an effective improvement of physical activity performance and motivation in sports participation. Moreover, augmented reality for training can be used as an easier and better method for home training sessions during and after the COVID-19 pandemic.

The article "Improvements of Physical Activity Performance and Motivation in Adult Men through Augmented Reality Approach: A Randomized Controlled Trial" was published in 2022. Journal: J Environ Public Health.

## Figures and Tables

**Figure 1:** Study flow diagram.

**Figure 2:** Group comparisons of the mean changes in muscle strength and muscle endurance.

**Figure 3:** Group comparisons of the mean changes in motivation, balance, and flexibility.

**Table 1:** General characteristics of respondents.

	MVFT group (*n* = 12)	TBT group (*n* = 12)	ART group (*n* = 12)	Control group (*n* = 12)
Age (years)	24.83 ± 3.099	23.83 ± 1.528	23.42 ± 1.564	23.92 ± 2.644
Height (cm)	175.75 ± 4.883	174.58 ± 7.267	174.50 ± 5.681	175.33 ± 4.793
Weight (kg)	76.17 ± 7.133	74.58 ± 7.342	75.92 ± 7.317	76.58 ± 7.128

mean ± standard deviation, MVFT: mirror visual feedback training, TBT: therapist-based training, ART: augmented reality-based training.

**Table 2:** Maximal isokinetic muscle strength muscle endurance within and between-group comparison.

Measurement	Group	Pretest	Posttest	*P*	Effect size
Knee extension strength (60°/s; Nm)	MVFT group	121.00 ± 52.14	129.25 ± 47.88^b^	0.036^*∗*^	0.158
	TBT group	165.42 ± 48.20	196.42 ± 47.21^c^	0.003^*∗*^	0.643
	ART group	177.08 ± 42.60	216.67 ± 32.91^b,d^	0.001^*∗*^	0.928
	Control group	137.17 ± 53.73	137.42 ± 53.45^c,d^	0.339	0.004

Knee extension endurance (Nm)	MVFT group	402.92 ± 127.41	407.00 ± 124.58^b^	0.012^*∗*^	0.032
	TBT group	410.25 ± 99.74	427.83 ± 112.15^c^	0.021^*∗*^	0.176
	ART group	409.08 ± 94.04	426.17 ± 86.24^b,d^	0.002^*∗*^	0.181
	Control group	410.92 ± 126.90	411.08 ± 127.00^c,d^	0.339	0.001

Knee flexion strength (60°/s; Nm)	MVFT group	161.25 ± 21.31	165.25 ± 22.46	0.026^*∗*^	0.187
	TBT group	161.42 ± 21.59	168.33 ± 28.09^c^	0.024^*∗*^	0.195
	ART group	162.33 ± 35.81	169.33 ± 33.00^d^	0.003^*∗*^	0.204
	Control group	162.08 ± 28.58	162.00 ± 28.51^c,d^	0.586	0.002

Knee flexion endurance (Nm)	MVFT group	402.58 ± 126.50	406.42 ± 124.45	0.032^*∗*^	0.030
	TBT group	408.58 ± 97.52	426.58 ± 111.54^c^	0.030^*∗*^	0.184
	ART group	408.00 ± 93.80	425.42 ± 84.91^d^	0.003^*∗*^	0.185
	Control group	405.75 ± 131.70	405.92 ± 131.81^c,d^	0.339	0.001

^*∗*^ *P* < 0.05, mean ± standard deviation; MVFT: mirror visual feedback training; TBT: therapist-based training; ART: augmented reality-based training; a: difference between MVFT and TBT; b: the difference between MVFT and ART; c: the difference between TBT and control group; d: the difference between ART and control group.

The article "Improvements of Physical Activity Performance and Motivation in Adult Men through Augmented Reality Approach: A Randomized Controlled Trial" was published in 2022. Journal: J Environ Public Health.

**Table 3:** Comparison of motivation, balance, and flexibility within group and between groups.

Measurement	Group	Pretest	Posttest	*P*	Effect size
Balance (cm)	MVFT group	97.06 ± 13.81	98.72 ± 13.79^a,b^	0.016^*∗*^	0.119
	TBT group	98.16 ± 5.96	103.46 ± 7.46^a,c^	0.000^*∗*^	1.888
	ART group	98.32 ± 6.06	105.87 ± 6.12^b,d^	0.000^*∗*^	1.245
	Control group	85.79 ± 16.80	86.91 ± 16.56^c,d^	0.111	0.066

Flexibility (cm)	MVFT group	3.50 ± 5.86	3.58 ± 4.85	0.931	0.014
	TBT group	3.07 ± 17.73	4.58 ± 14.27	0.269	0.084
	ART group	3.50 ± 13.24	4.83 ± 14.94	0.132	0.100
	Control group	3.08 ± 8.72	2.91 ± 8.71	0.638	0.019

Intrinsic motivation (points)	MVFT group	79.75 ± 2.95	81.33 ± 2.70	0.029^*∗*^	0.535
	TBT group	78.17 ± 4.23	80.00 ± 5.00	0.017^*∗*^	0.432
	ART group	84.00 ± 2.37	86.33 ± 4.09	0.012^*∗*^	0.982
	Control group	80.42 ± 2.10	80.75 ± 2.13	0.305	0.157

^*∗*^ *P* < 0.05, mean ± standard deviation; MVFT: mirror visual feedback training; TBT: therapist-based training; ART: augmented reality-based training; a: difference between MVFT and TBT; b: the difference between MVFT and ART; c: the difference between TBT and control group; d: the difference between ART and control group.

## Data Availability

The datasets used to support the findings of this study are available from the corresponding author on reasonable request.
